# Implementation of CT Image Segmentation Based on an Image Segmentation Algorithm

This article has been retracted.

**DOI:** 10.1155/2022/2047537

**Published:** 2022-10-12

**Authors:** Lingli Shen

**Affiliations:** Shanghai East Hospital, Shanghai, China

## Abstract

With the increasingly important role of image segmentation in the field of computed tomography (CT) image segmentation, the requirements for image segmentation technology in related industries are constantly improving. When the hardware resources can fully meet the needs of the fast and high-precision image segmentation program system, the main means of how to improve the image segmentation effect is to improve the related algorithms. Therefore, this study has proposed a combination of genetic algorithm (GA) and Great Law (OTSU) algorithm to form an image segmentation algorithm-immune genetic algorithm (IGA) algorithm. The algorithm has improved the segmentation accuracy and efficiency of the original algorithm, which is beneficial to the more accurate results of CT image segmentation. The experimental results in this study have shown that the operating efficiency of the OTSU segmentation algorithm is up to 75%. The operating efficiency of the GA algorithm is up to 78%. The operating efficiency of the IGA algorithm is up to 92%. In terms of operating efficiency, the OTSU segmentation algorithm has more advantages. In terms of segmentation accuracy, the highest accuracy rate of OTSU segmentation algorithm is 45%. The accuracy of the GA algorithm is 80%. The highest accuracy of the IGA algorithm is 97%. The IGA algorithm is more powerful in terms of operating efficiency and accuracy. Therefore, the application of the IGA algorithm to CT image segmentation is beneficial to doctors to better judge the lesions and improve the diagnosis rate.

## 1. Introduction

With the improvement of people's quality of life, the society's demand for the medical industry is increasing. In order to simplify the work of doctors' diagnosis, computer-aided diagnosis technology has been widely researched and developed. The abdomen is one of the parts of the human body with many tissues and organs, the most complex structure and high incidence. Therefore, the diagnostic technology of abdominal medical computed tomography (CT) images has important research value. How to accurately locate and segment organs and tissues from medical images is an important prerequisite for the realization of abdominal medical diagnosis technology. The area of medical imaging underwent a revolution when CT technology was developed in the early 1970s. Medical imaging shows the structure and density of the internal tissues and organs of the human body in the form of images, which is used by the diagnosing physicians to judge according to the information provided by the images, so as to evaluate the health status of the human body. In addition, radiation CT, digital stereography, ultrasound imaging, magnetic resonance imaging, and modern medical diagnosis have undergone major changes due to computer and medical image processing techniques that have laid the foundation for the development of these imaging techniques.

Technology for medical diagnosis and treatment has advanced significantly, and several novel CT image segmentations are suitable for clinical diagnosis and therapy. Additionally, the data generated by combining several imaging modalities can reach complementarity and offer a solid scientific foundation for biomedical research and clinical diagnostics. As a result, CT image segmentation technology has received a lot of attention and has advanced quickly. Medical image processing has gotten more and more attention from academics as CT image segmentation technology has continued to advance. The most important technique for processing and analyzing medical images is CT image segmentation. In image medicine, picture segmentation is becoming more and more crucial. Image segmentation is a crucial tool for removing quantitative data from specific tissues in images. It is also a necessary step before visualization and is applied in many different fields. The innovation of this study is that the basic algorithm based on the image segmentation algorithm is proposed, and the image segmentation algorithm is improved based on the genetic algorithm (GA). Experiments have proved that the proposed algorithm is meaningful.

## 2. Related Work

One of the medical technology development fields with the quickest growth rate over the past 20 years is medical CT imaging. This technology enables clinicians to observe the internal lesions of the human body more directly and clearly, and the diagnosis rate is also improved. Suzuki et al. has found that one needs to evaluate not only the value of mechanical properties but also the degree of damage in order to maintain concrete structures effectively. They have suggested the use of X-ray CT for damage estimation of concrete [1]. Ha et al. has found that the attribution of reduced intracranial cerebrospinal fluid (CSF) volume in patients with mass-occupying masses is associated with reduced cerebral perfusion pressure and subsequent cerebral ischemia. Their aim was to assess the ratio of CSF volume to brain volume using CT images [2]. Dijk et al. has found that CT images currently used to predict moderate-to-severe xerostomia in advanced post-radiotherapy patients are highly accurate. They have investigated 249 patients with head and neck cancer who received definitive CT scans and radiation therapy [3]. Zorn et al. has been designed to build the learning curve associated with achieving standardized post-processing for radiographer students. To discuss their interests, each student has repeated 2 of the 15 CT post-processing protocols. They have also assessed each student's achievement accuracy at each repetition. Results have shown that the learning rates for the two protocols are 63% and 56%, respectively [4]. Li et al. has found that norm regularization has attracted attention in computerized CT scan image reconstruction. CT image gradients have provided a measure of image gradient sparsity for reconstructing images from finite projection data in CT and have effectively addressed optimization problems [5]. Scholars have seen that CT images are not only used in the medical field, but also used in various fields to a certain extent, which also shows that CT images have made great progress. However, applying image segmentation to it would make it more effective.

Medical image segmentation is the process of dividing an image into several regions according to the similarity within the region and the difference between the regions. How to separate relevant structures and regions of interest from images is the first problem to be solved by image analysis and recognition, and it is also a bottleneck that limits the development and application of other related technologies in medical image processing. Chen et al. has discovered that deep learning can be used to solve semantic image segmentation, and they have highlighted the great promise of convolutions using upsampling filters. As a powerful tool in dense prediction tasks, convolution can control the resolution in deep convolutional neural networks [6]. Mariano et al. has proposed an image segmentation framework based on maximum likelihood estimation, which has been generated by sampling with different likelihood functions. They have also proposed efficient segmentation methods capable of dealing with textured images [7]. A fresh heterogeneous neural network model for image segmentation has been put out by Yang et al. The image is divided into many sections based on the gray level, and different neurons correlate to various parameters. The outcomes have proven that the suggested segmentation strategy is successful and efficient [8]. Mean shift, a widely used algorithm for multi-feature segmentation, has been discovered by Cuevas et al. to be more effective than one-dimensional feature methods. They have developed a novel, competitive segmentation technique for grayscale images that has already taken into account the local variance and grayscale value of each pixel [9]. Scholars have proposed that neural network can be used in image segmentation to improve the accuracy and efficiency of image segmentation, and it has been considered that image segmentation can achieve important development in various fields. However, scholars have not presented specific cases to prove this point.

## 3. CT Image Segmentation Method Based on Image Segmentation

With the emergence of computer-aided diagnosis and medical images for clinical auxiliary diagnosis, the diagnosis efficiency of clinicians has been greatly improved, and this field has attracted more and more attention of researchers. In the realm of image processing and computer vision, picture segmentation is a crucial component and a challenge [10–12]. The technology and procedure of dividing an image into sections with various properties and extracting items of interest is known as image segmentation. This is both a fundamental computer vision technique as well as a crucial step from image processing to image analysis. It makes it possible to grasp feature extraction and parameter measurement targets at a higher level of picture analysis. Research on image segmentation techniques is crucial since the subsequent processing directly depends on how accurate the segmentation results are.

CT is less effective for soft tissue contrast imaging, but with high density resolution, it can clearly display bone, muscle, and organ information [13]. CT scans a certain part of the human body one by one with a highly sensitive detector. It has the characteristics of fast scanning time and clear image. Each scan needs to inject a contrast agent, which is a scan image with radioactive radiation, the cheapest price, and the most widely used medical imaging. Magnetic resonance imaging is an imaging based on radio waves and has the highest spatial resolution. It has better resolution for soft tissue (cranial structure) in the human body and can achieve functional imaging. However, it has low sensitivity, long image acquisition time, and moderate price [14]. However, since only labeled CT images are currently published in the field of liver segmentation, CT imaging is used under data constraints. CT imaging is shown in Figure 1.

As shown in Figure 1, the cross-sectional images obtained by CT scanning can also be reorganized and reconstructed by computer software to obtain multi-plane cross-sectional images such as sagittal and coronal planes required for diagnosis. The CT medical device scanning apparatus sends X-rays into the body's numerous tissues and organs, returning varying response values depending on the organs and tissues. A particular interface function is needed to read medical data in DICOM format files, which are the data output from CT medical equipment, in order to load images [15]. Diverse CT scanning imaging equipment is employed as a result of the diversity of CT medical scanning equipment, and the gray value range of the CT image produced by the corresponding scanning is also different [16]. Setting the appropriate window width and window level values for the CT image is required in order to display the pixel range truncation and display the DICOM data image appropriately. The values within the window width are mapped to the values between [0, 255] through linear transformation, defined as formula (1):

(1) $$\begin{array}{c} G\left(V\right)=\left(\frac{V-\left(C-0.5\right)}{W-1}+0.5\right)\times 255.0, \end{array}$$

where 255.0 is the original image data, *W* is the window width value, *C* is the window level value, and *G*(*V*) is the converted pixel value.

### 3.1. Image Segmentation Based on GA

In the 1960s, some scholars proposed an operation that conformed to the hardware conditions at that time. The most obvious disadvantage of this automatic threshold selection method based on gray histogram is that it needs to measure the ratio of the image segmentation target to the whole image before segmentation. The artificial measurement method results in a very low repetition rate of this segmentation operation, known as the P-tile method [17]. The P-tile algorithm is an automatic threshold selection algorithm based on gray histogram statistics, which needs to be based on certain prior conditions. The schematic diagram of image segmentation is shown in Figure 2.

As it can be seen from Figure 2, the existing image segmentation methods are mainly divided into the following categories: threshold-based segmentation methods, region-based segmentation methods, edge-based segmentation methods, and specific theory-based segmentation methods. In the 1980s, there was a theory based on the extraction of full-image pixel information combined with mathematical methods to obtain the best fitness. The reason why this theory is not widely accepted is that its noise reduction is not ideal and the workload is large [18]. It is expressed as formula (2):

(2) $$\begin{array}{c} w_{0}\left(s,t\right)=\overset{s}{\underset{i=0}{\sum }}\overset{t}{\underset{j=0}{\sum }}P_{i,j}. \end{array}$$

The OTSU algorithm is a preliminary progress in the processing of pixel extraction gray histogram in image segmentation. After obtaining the gray level information of the histogram, the optimal value is obtained by comparing the algorithm, and the important operator of image segmentation—threshold value is determined from this [19]. OTSU is a commonly used algorithm in threshold segmentation, which can automatically generate the best segmentation threshold based on images. The core idea of OTSU is to maximize the variance between classes. The OTSU algorithm does not need any manual evaluation work in the early stage, but the process of obtaining the optimal solution requires a huge number of operations. If this contrast is defined as a matrix, the important variable of the operational formula is as follows formula (3):

(3) $$\begin{array}{c} \mu_{i}\left(s,t\right)=\overset{s}{\underset{i=0}{\sum }}\overset{t}{\underset{j=0}{\sum }}iP_{i}. \end{array}$$

When the variance value is formula (4), the minimum gray value to the maximum gray value are involved.

(4) $$\begin{array}{c} \mu_{j}\left(s,t\right)=\overset{s}{\underset{i=0}{\sum }}\overset{t}{\underset{j=0}{\sum }}jP_{j}. \end{array}$$

From the analysis of the OTSU algorithm, it can be known that *w*_0_(*s*, *t*), *μ*_*i*_(*s*, *t*), and *μ*_*j*_(*s*, *t*) should not only accumulate and sum, but also incorporate all the summation results into all (*s*, *t*). After the summation and merging of huge data, this operation is very complex and time-consuming [20].

In order to reduce the time complexity, some scholars use efficient hardware equipment with specific calculation principles to calculate the OTSU algorithm, and the effect is also not very ideal [21]. Moreover, once the gray value distribution of the segmented source image is chaotic, and the normal extreme value cannot be obtained, the high-precision segmentation result cannot be obtained by using the OTSU method.

With the continuous in-depth research of previous scholars, a theoretical idea that analyzes the solution of image segmentation operators with evolutionary theory has emerged, that is, the early GA is applied to the image segmentation threshold [22]. Compared with some conventional optimization algorithms, GA can usually obtain better optimization results faster. GAs have been widely used in combinatorial optimization, machine learning, signal processing, adaptive control, and artificial life. The basic idea of GA is to mathematically describe Darwin's theory of biological evolution, so as to abstract it for modeling and form a traversal algorithm. GA has strong and comprehensive parallelism in calculation, which can reasonably prevent premature convergence, and parallelism can be effectively hidden or contained in the process of crossover and mutation calculation. The noise processing method is relatively mild, and has the advantages of certain elimination and identification measures and reasonable calculation speed. The structure diagram of the GA is shown in Figure 3.

As shown in Figure 3, GAs generally do not need other external information in the process of search evolution, and only use evaluation functions to evaluate the pros and cons of individuals or solutions, thus serving as the basis for subsequent genetic operations. Using GA combined with the idea of region segmentation technology in image segmentation theory, the image to be segmented can be segmented and modeled. The optimal threshold can be obtained by performing modeling operations in the model, and this threshold is the segmentation result that can be obtained in the image area that needs to be segmented. Because mathematical modeling is very difficult, how to use the mathematical model to obtain the best threshold to obtain the ideal segmentation effect has always been the difficulty of image processing technology, especially image segmentation technology. In this study, it tries to combine the improved GA optimization method with the maximum inter-class variance method improved by this study, and gives full play to the advantages of each method to achieve a good segmentation effect. In the GA calculation, in order to make the algorithm retain the individual's good genes, the adaptive GA can be used to adjust the traditional GA adaptive degree problem. Let the crossover operator be *P*_c_, if they need to be adjusted automatically with the fitness, there is formula (5):

(5) $$\begin{array}{c} P_{c}=\left\{\begin{array}{c} \frac{k_{1}\left(f_{\max}-f^{\prime }\right)}{f_{\max}-f_{\text{avg}}},f\geq f_{\text{avg}}\\ k_{2},f<f_{\text{avg}} \end{array}\right.. \end{array}$$

Among them, *f*_max_ is the largest fitness value in a specific group. *f*_avg_ is the average fitness value of each generation of the group. *f*′ is the larger fitness value in the operator that requires crossover operation. *f* is the general fitness value that requires mutation operation. These coefficients are often excellent seeds selected in the early stage of evolution, and they remain unchanged when other seeds evolve, thus shielding their own evolution and causing the calculus to fall into a local optimum.

Adding two variables *f*_max_ is the maximum mutation probability and *P*_*c*1_ is the maximum crossover probability. It is expressed as formula (6):

(6) $$\begin{array}{c} P_{c}=\left\{\begin{array}{c} P_{c1}\cdot e^{f-f_{\text{avg}}/f_{\max}-f_{\text{avg}}},f\geq f_{\text{avg}}\\ P_{c1},f<f_{\text{avg}} \end{array}\right.. \end{array}$$

The so-called activation function is the function running on the neurons of the artificial neural network, which is responsible for mapping the input of the neuron to the output. In a neural network, there is a neuron activation function sigmoid that can balance linear and nonlinear behavior, and its expression is as shown in formula (7).

(7) $$\begin{array}{c} \phi \left(v\right)=\frac{1}{1+\exp\left(-av\right)}. \end{array}$$

Using the sigmoid function, the two operators of crossover probability and mutation probability can be improved to ensure that the curve is always in a smooth state at *f*.

### 3.2. Image Segmentation Based on Improved GA-IGA Image Segmentation Method

When performing image segmentation, how to choose the most suitable grayscale threshold for this segmentation in the grayscale image is the key to effectively separating the target image from the background image. The grayscale threshold is to divide all the brightness values in the image into two categories higher than the threshold and lower than the threshold according to the specified brightness value (i.e., the threshold). If the background information points are mistakenly divided into target information during the calculation process, the segmentation effect may be deviated. Therefore, it is necessary to use the algorithm to keep the target away from the background, that is, the larger the class spacing between the two, the noise would be shielded, so that the segmented target would be more accurate.

The binarization of the image is to set the gray value of the pixels on the image to 0 or 255, that is, the entire image presents an obvious visual effect of only black and white. At the same time, after the image is binarized, the distance between each piece of pixel information and the image center information is opposite. The closer the distance is, the better the cohesion of the pixels between each category is. This idea uses the average variance of the two types to express as formula (8):

(8) $$\begin{array}{c} {\sigma_{0}}^{2}\left(t\right)=\frac{1}{w_{0}\left(t\right)}\underset{0\leq t}{\sum }{\left(i=\mu_{0}\left(t\right)\right)}^{2}p\left(i\right). \end{array}$$

In this formula, *μ*_0_(*t*) and *w*_0_(*t*) represent the target gray value and the background gray value, respectively, and t is the gray threshold. Through variance operation, it can be obtained that the more uniform the distribution of pixels within the class, the better the cohesion between individuals, so that the target and the back are easier to distinguish.

In order to solve the problems of class cohesion and the distance between the target and the background class, this study improves the threshold value based on the basic OTSU method is defined as formula (9):

(9) $$\begin{array}{c} G\left(t\right)=\frac{w_{0}\left(t\right)w_{1}\left(t\right){\left(\mu_{0}\left(t\right)-\mu_{1}\left(t\right)\right)}^{2}}{\sigma_{0}^{2}+\sigma_{1}^{2}}. \end{array}$$

When *G*(*t*) takes the maximum value, the corresponding gray level is the obtained optimal threshold value Th. It is expressed as formula (10):

(10) $$\begin{array}{c} \text{Th}=\arg\max\left[G\left(t\right)\right]. \end{array}$$

*G*(*t*) and *μ*_1_(*t*) represent the target gray value and the background gray value, respectively, and according to the optimal gray threshold *t* obtained by the formula, it can be obtained by formula (11):

(11) $$\begin{array}{c} d^{2}\left(t\right)={\left(u_{0}\left(t\right)-u_{1}\left(t\right)\right)}^{2}. \end{array}$$

In order to obtain the optimal solution of *d*^2^(*t*), the optimization of *d*^2^(*t*) can be realized by combining the evolution process of GA and this kind of GA is called improved GA IGA. The algorithm is realized by the combination of GA and OTSU. A functional is a mapping from functions to numbers. An operator is a mapping from functions to functions. The improved IGA mainly realizes nonlinear adjustment in the crossover and mutation operators. The operator function is expressed as formula (12):

(12) $$\begin{array}{c} P_{c}=\left\{\begin{array}{c} \frac{p_{c\max}-p_{c\min}}{1+\exp\left(A\left(2\left(f^{\prime }-f\right)/f_{\max}-f-1\right)\right)}\\ p_{c\min},f^{\prime }\leq f \end{array}\right.f^{\prime }>f. \end{array}$$

In this study, the classification error is used to evaluate the pros and cons of the algorithm, which is usually ME ∈ [0, 1] for the convenience of analysis. The calculation formula for misclassification is expressed as formula (13):

(13) $$\begin{array}{c} \text{ME}=1-\frac{\left|G_{0}\cap G\right|+\left|F_{0}\cap F\right|}{\left|\left|G_{0}\right|+\left|F_{0}\right|\right|}. \end{array}$$

where *G*_0_ and *F*_0_ represent the target and background areas in the original image when ideally segmented, respectively.

### 3.3. CT Image Segmentation Based on IGA Algorithm

If the input abdominal CT scan sequence traverses the cross-sectional slice image sequence along the vertical axis from the top of the liver to the right lung lobe, the shape and area of the liver tissue area in the slice image would gradually become larger. This method is mainly based on the consistency and similarity of organs and tissues between CT image sequences. The human CT image segmentation is shown in Figure 4.

Figure 4(a) is the segmentation of the CT image before scanning, and Figure 4(b) is the segmentation of the CT image after scanning. The third layer of the whole sequence was selected as the initial slice layer. After analysis, the liver tissue in this slice had a larger area, a clear edge, and a distinct degree of distinction in the shape and outline of the liver tissue. Only a small amount of initial manual labeling is required to obtain accurate initial liver tissue segmentation contours. Interactive image segmentation means that the user first specifies part of the foreground and part of the background of the image by some interactive means, and then the algorithm uses the user's input as the segmentation constraints to automatically calculate the optimal segmentation that meets the constraints. In this study, the liver tissue segmentation of the initial slice image adopts the interactive graph cut algorithm, and the label value vector of all pixels on the image is defined as Formula (14):

(14) $$\begin{array}{c} L^{n_{0}}=\left(l_{1}^{n_{0}},\cdots ,l_{i}^{n_{0}},\cdots ,l_{I}^{n_{0}}\right). \end{array}$$

Since it is currently a binary classification problem, the label value *l*_*i*_^*n*_0_^ ∈ {0, 1} represents the label value of the *i*th pixel in the initial slice layer *l*_*i*_^*n*_0_^. The label value of 0 represents the background, otherwise it is the foreground. The segmentation energy function of the initial slice is defined as formula (15):

(15) $$\begin{array}{c} E\left(L^{n_{0}}\right)=\underset{i\in I}{\sum }R\left(l_{1}^{n_{0}}\right)+\lambda_{0}*\underset{\left(i,j\right)\in E}{\sum }B\left(l_{i}^{n_{0}},l_{j}^{n_{0}}\right). \end{array}$$

Among them, pixels *i* and *j* are adjacent pixels connected by weights. *λ*_0_ is a constant coefficient, which measures the proportion of boundary items and area items.

The area item *R*(*l*_1_^*n*_0_^) represents the penalty item with the label value *l*_1_^*n*_0_^ assigned to 0 and 1, respectively. If the gray value of the pixel *i* is *g*_*i*_, the formula of the area item is defined as formula (16):

(16) $$\begin{array}{c} R\left(l_{i}^{n_{0}}=0\right)=-\text{In}\left(P_{fg}\left(g_{i}\right)\right). \end{array}$$

Grayscale values refer to the color value of each object when converting a grayscale object to RGB. The relationship between white and black is divided into several levels according to the logarithmic relationship, which is called “gray level.” When the pixel *i* is marked as 0, the region item of the pixel is the negative logarithm of the gray value of the pixel in the foreground gray histogram, and it is the opposite when it is marked as the foreground 1. The region item intuitively reflects that the pixel *i* is marked as a penalty item and they have corresponding labels.

The boundary *B*(*l*_*i*_^*n*_0_^, *l*_*j*_^*n*_0_^) indicates that adjacent pixels *i* and *j* are penalized with different label values. The specific calculation formula is as shown in formula (17).

(17) $$\begin{array}{c} B\left(l_{i}^{n_{0}},l_{j}^{n_{0}}\right)=\delta \left(l_{i}^{n_{0}},l_{j}^{n_{0}}\right)\times \frac{1}{\left(g_{i},g_{j}\right)+1}. \end{array}$$

Combining the above formulas to define the value of the label vector, the global optimal liver segmentation result of the initial layer is obtained by constructing the minimization solution formula, as shown in formula (18).

(18) $$\begin{array}{c} L^{*n_{0}}=\arg\min E\left(L^{n_{0}}\right). \end{array}$$

The abdominal region of the human body is one of the parts with the most tissues and organs, the most complex structure and a high incidence of disease. With the development and popularization of computers in various industries, computer-aided disease diagnosis technology is becoming more and more mature. However, abdominal CT scan images are easily affected by the motion and noise of the tissues affecting the body and the low resolution of the equipment itself, which brings great challenges to the correct segmentation of tissues and organs in CT scan images. The improved image segmentation algorithm-IGA algorithm proposed in this study improves the segmentation accuracy and efficiency of traditional image segmentation algorithms.

## 4. Experiment of CT Image Segmentation

### 4.1. Experiments on the Segmentation Effect of Three Image Segmentation Algorithms

All the algorithms in the experiment simulation of the algorithm in this study are completed on the notebook, and the CPU and running memory are 2.4 GHz and 4 GB RAM, respectively. The algorithm implementation software is MATLAB 2016a. In order to verify the efficiency of the proposed algorithm, program model experiments are carried out on the OTSU segmentation algorithm, the GA algorithm, and the IGA algorithm, respectively. In order to highlight the practicality, the images selected in this part are several unconstrained images annotated.

The experiment tests the calculation time of OTSU segmentation algorithm, GA algorithm, and IGA algorithm, and the number of experiments is five times. The thresholds and time-consuming conditions of the three segmentation methods are shown in Table 1.

As shown in Table 1, it can be seen that the IGA algorithm saves one-third of the time compared to the OTSU method, and is nearly 5 ms faster than the GA algorithm with the advantage of fast operation speed. In terms of the accuracy of the threshold, although it is not as stable as the OTSU segmentation algorithm, the change of the threshold is controlled within 2 pixels. It shows that IGA is more real-time in the feedback of calculation results. According to human eye observation, the segmentation range of OTSU segmentation algorithm, GA algorithm, and IGA algorithm is slightly different. The two GAs are slightly better than the OTSU method, and the IGA algorithm is more accurate. The comparison of the segmentation results shows that the IGA algorithm also has certain advantages in computing accuracy when segmenting complex image targets.

In order to compare the accuracy of the three algorithms in the segmentation edge more accurately, the segmentation experiment is continued. This study does not continue to segment the head target, but selects the human body contour as the segmentation target after the image is grayed. On this basis, the accuracy of the head results after segmentation is compared. The results are shown in Table 2.

As shown in Table 2, since the image is segmented after grayscale, it can be found that the thresholds of the three algorithms are relatively stable, and the OTSU method is the most accurate but has poor real-time performance. GA is still a short time, but the threshold changes are active, around 4 pixels. The threshold of IGA changes within 2 pixels, but the time is about four times faster than that of OTSU. It is more stable in both time and segmentation accuracy. It is shown in Figure 5.

Figure 5(a) illustrates that the head's contour is subject to errors if the OTSU method is used to process the image because the target contour is clearer but the interference is poor. The outcome of segmentation using the GA approach is displayed in Figure 5(b). Although GA's contour processing is less thorough than OTSU's, the primary objective is still evident. It displays the versatility and global search benefits of the GA algorithm. The IGA algorithm can see that the human head target in the segmentation area is relatively complete and the segmentation accuracy is relatively high.

The three algorithms of GA, OTSU, and IGA are calculated through 100 generations of evolution, and the adaptive degrees are obtained as shown in Figure 6.

As shown in Figure 6, compared with GA, IGA and OTSU have a better adaptive degree in the evolution process, and the strong ability to get rid of them can also avoid local precociousness. Only IGA can obtain the optimal solution in the 20th generation, although there is an oscillation divergence in the middle. But because of its strong adaptive ability, it quickly returned to the normal computing state. From the above curves, it can be seen that the adaptability and robustness of IGA are better than GA and OTSU.

It is well known that usually if an algorithm uses double adaptation, it may lead to contradictions in the internal mechanism of the algorithm. In order to eliminate this contradictory effect, a large number of parameter selection experiments are hereby done. It is shown in Figure 7.

As can be seen from Figure 7(a), for different types of test images, the proposed algorithm obviously has better segmentation quality. The segmentation result has a higher signal-to-noise ratio. Compared with other algorithms, the segmented image has clearer target information, and the segmented target image has a clearer outline. The segmented outline information, for instance, is more evident than other algorithms, as the graphic illustrates.  Figure 7(b) demonstrates that, despite of not appearing to be very obvious, a deeper examination of the segmentation outcomes produced by the suggested algorithm is usually preferable. As a result, when compared to existing algorithms, the suggested technique may yield excellent segmentation results for a variety of image formats, demonstrating a wider range of applications.

### 4.2. Experiments on the Efficiency of the Three Algorithms

Although image threshold segmentation has been studied for many years and various algorithms emerge in an endless stream, the problem of image threshold segmentation becomes more and more complicated due to the variety of images and the sources of images. The existing algorithms are basically specific algorithms that can only solve some specific images, which is very limited. Tables 3 and 4 show the classification errors of the three algorithms in the study and the running time of the algorithms after segmenting the five medical images in the experiment:

As shown in Tables 3 and 4, compared with other different algorithms, the IGA algorithm proposed in this study not only reduces the misclassification rate greatly. Moreover, the overall running time is the shortest, and in most cases a satisfactory segmentation threshold can be achieved with fewer iteration steps. Therefore, whether it is an intuitive evaluation standard or an objective evaluation standard, the algorithm proposed in this study has a good segmentation effect, especially in the processing of medical CT images with relatively less complex details.

The method in this study is utilized to carry out segmentation studies on group data to confirm the efficacy of the method. The experimental data comes from lung CT images of the First Affiliated Hospital of a university. There are 10 groups of normal images, and the nodule size is 4–30 mm. Each set of data contains 35–45 frames, and the analysis of the obtained segmentation results are shown in Figure 8.

Figure 8(a)illustrates how far the OTSU method's segmentation effect differs from the manual method's segmentation effect.  Figure 8(b) illustrates how the segmentation impact of the GA approach is superior to that of Figure 8(a). Manual segmentation still has a significantly worse impact than automatic segmentation, though.  Figure 8(c) shows that the IGA method is more similar to the results of manual segmentation and can obtain the complete lung parenchyma edge, avoiding the omission of lung nodules. The proposed method can effectively segment the lung parenchyma from normal and diseased lung images. The segmentation results obtained by applying the method in this study to the left and right lungs are very similar to the results obtained by the clinicians' manual segmentation, and the obtained segmentation results are satisfactory to the clinicians.

Although this study chooses the OTSU method as the main algorithm for calculating the threshold based on theory and experiments, the variability of important links, such as selection, crossover, and mutation during the operation of the algorithm may lead to other algorithms participating in the improvement. It is also an important direction for future research that the population has better self-adaptability to ensure excellent robustness during global evolution.

## 5. Conclusions

Image segmentation is not only one of the main techniques of image processing, but also one of the key techniques of object recognition and object detection. The main idea is to separate the target information from the background information. Then the target information is marked and identified through a certain algorithm. Finally, the target information is extracted from the image. In this study, the traditional image segmentation method has been improved, and an image segmentation method has been formed. In order to improve the segmentation accuracy, the GA is avoided to fall into a local optimum because of precociousness. On the basis of improving the traditional GA and optimizing the single-dimensional OTSU method, this study uses the different characteristics of the two algorithms to form an improved algorithm IGA. Through experiments, it is found that the improved algorithm shows advantages in terms of calculation time, computational complexity, and segmentation effect. It is especially suitable for segmentation of CT images. Although the IGA proposed in this study has certain advantages over the algorithm before the improvement in the test results, in the experiment, the unscientific sample selection would cause obstacles to the operation. The main research direction in the future is still to be attributed to the optimization and selection of control parameters.

## Figures and Tables

**Figure 1:** CT imaging.

**Figure 2:** Schematic diagram of image segmentation.

**Figure 3:** The structure diagram of the genetic algorithm.

**Figure 4:** Human CT image segmentation. (a) Before scanning. (b) After scanning.

**Figure 5:** Comparison of the effects of three methods for processing images. (a) Comparison of the effects of the three methods for processing the contour of the image target. (b) Comparison of the effects of the three methods for eliminating interference.

**Figure 6:** Adaptability of the three methods.

**Figure 7:** Segmentation effect of the three algorithms in the case of different image clarity. (a) The segmentation effect of the three algorithms when the image is clear. (b) The segmentation effect of the three algorithms when the image is blurred.

**Figure 8:** Comparison of the proximity of three methods of lung CT image segmentation and manual segmentation. (a) The proximity comparison between the segmentation effect of the OTSU method and the manual segmentation. (b) The proximity comparison between the segmentation effect of the GA method and the manual segmentation. (c) The proximity comparison between the segmentation effect of the IGA method and the manual segmentation.

**Table 1:** Thresholds and time-consuming conditions of the three segmentation methods.

Number of experiments		1	2	3	4	5
GA	Image threshold	115	115	115	115	115
	Time (ms)	28.21	21.46	26.03	26.07	26.15
OTSU	Image threshold	130	130	130	130	130
	Time (ms)	13.37	14.28	14.52	14.43	14.55
IGA	Image threshold	132	132	132	132	132
	Time (ms)	10.02	9.15	9.53	9.87	9.66

**Table 2:** Efficiency of three algorithms for segmenting edges.

Number of experiments		1	2	3	4	5
GA	Image threshold	70	70	70	70	70
	Time (%)	78	70	76	77	76
OTSU	Image threshold	85	85	85	85	85
	Time (%)	75	72	71	75	70
IGA	Image threshold	90	90	90	90	90
	Time (%)	92	90	91	88	87

**Table 3:** Classification errors after segmentation of medical images.

Images	GA (%)	OTSU (%)	IGA (%)
1	27	12	2
2	20	10	5
3	22	16	4
4	38	18	8
5	21	15	7

**Table 4:** Medical image segmentation running time.

Images	GA (s)	OTSU (s)	IGA (s)
1	0.97	0.68	0.21
2	0.90	0.75	0.26
3	0.93	0.72	0.23
4	0.92	0.73	0.27
5	0.95	0.71	0.24

## Data Availability

Data sharing not applicable to this article as no datasets were generated or analyzed during the current study.
